The article "Effects of the Concept of Fast-Track Surgery Combined with Empathic Nursing on Perioperative Complication Prevention and Postoperative Recovery of Gynecological Malignant Tumor Patients" was retracted in 2023. Reasons: signs of a paper mill; suspected computer-generated content; unreliable results or conclusions; concerns about the data.

# Effects of the Concept of Fast-Track Surgery Combined with Empathic Nursing on Perioperative Complication Prevention and Postoperative Recovery of Gynecological Malignant Tumor Patients

**DOI:** 10.1155/2022/4381297

**Published:** 2022-07-31

**Authors:** Xiaoyan Duan, Miaomiao Liu, Pei Wang

**Affiliations:** ^1^Department of Gynecology, Hebei General Hospital, Shijiazhuang, Hebei 050051, China; ^2^Department of Oncology, Hebei General Hospital, Shijiazhuang, Hebei 050051, China

## Abstract

**Objective:**

This study is aimed at exploring the effects of the concept of fast-track surgery (FTS) combined with empathic nursing on perioperative complication prevention and postoperative recovery of gynecological malignant tumor patients.

**Methods:**

A total of 180 patients with gynecological malignant tumor treated by surgery in our hospital from September 2018 to October 2021 were randomly divided into three groups: group A, group B, and group C, with 60 patients in each group. Group C was given conventional nursing intervention, group B was given FTS intervention, and group A was given FTS intervention combined with empathic care. Psychological stress state (systolic blood pressure, diastolic blood pressure, and heart rate), postoperative recovery indicators (time of first anal exhaust, time of first defecation, time of getting out of bed, and length of postoperative hospital stay), postoperative complications, and psychological state (Self-Rating Anxiety Scale (SAS) and Self-Rating Depression Scale (SDS)) levels of patients in the three groups were compared.

**Results:**

Systolic blood pressure, diastolic blood pressure, and heart rate in group A were lower than those in group B, and those in group B were lower than those in group C (all *P* < 0.05). The time of first anal exhaust, time of first defecation, time of getting out of bed, and postoperative hospital stay in groups A and B were shorter than those in group C (all *P* < 0.05).The incidence of postoperative complications in groups A and B was 8.33% and 8.33%, respectively, lower than 23.33% in group C (both *P* < 0.05). SAS and SDS scores of group A were lower than those of groups B and C after intervention (all *P* < 0.05).

**Conclusion:**

The concept of FTS combined with empathic nursing is beneficial to reduce the stress response of patients with gynecological malignant tumor before surgery, reduce the risk of postoperative complications, improve patients' mood, and speed up the rehabilitation process of patients.

## 1. Introduction

Gynecological malignant tumors seriously threaten women's physical and mental health. Clinically common gynecological malignant tumors mainly include cervical cancer, ovarian cancer, and endometrial cancer, among which cervical cancer ranks first among all kinds of gynecological malignant tumors [1]. After diagnosis of gynecological malignant tumor, patients often need to receive comprehensive treatment such as surgery and multiple chemoradiotherapy, which brings great psychological and physiological pain to patients [2]. Clinically, due to the lack of disease-related cognition, patients often have a strong sense of uncertainty about the outcome of the disease [3, 4]. Meanwhile, as a physiological stress event, surgery may induce patients to develop a series of adverse psychological conditions such as anxiety and depression, which is not conducive to postoperative recovery. FTS integrates and applies a series of evidences based on evidence-based medicine, in order to effectively reduce the surgical stress response of patients, accelerate the process of postoperative rehabilitation, reduce the risk of postoperative complications, and improve the prognosis of patients [5]. At present, the concept of FTS has been widely used in colorectal surgery [6] and orthopedics [7]. Pache et al. [8] applied the concept of FTS to patients undergoing benign transabdominal gynecological surgery and confirmed that this concept could effectively reduce surgical stress response and promote postoperative recovery. In recent years, with the change of medical model and the development of psychosomatic medicine, people gradually realize that physical health and mental health are equally important. The elderly are more vulnerable. When told to have a malignant tumor and have an operation, they will be extremely anxious or depressed. If the medical staff do not pay attention to the mental health of patients, it may lead to the failure of surgery. Due to the special significance of uterus and ovary for women, compared with other malignant tumors, patients may bear greater psychological pressure but also bring heavy burden to society and family, affecting the quality of life of patients [9]. The concept of empathy originated in psychology, and empathy is a core technology treatment. After being introduced to medical nursing, empathic nursing has gradually become one of the core contents of psychological nursing. Empathy nursing considers problems from the perspective of patients, patiently listens to the real feelings of patients, understands the inner world of patients, and adopts targeted nursing services to guide patients out of psychological misunderstandings [10, 11]. Empathy has been widely used in clinical nursing, but rarely in gynecological malignant tumors. In this study, the concept of FTS combined with empathic nursing was applied to the perioperative nursing of gynecological malignant tumors, and its application value was expounded by comparing with conventional nursing intervention. The report is as follows.

The article "Effects of the Concept of Fast-Track Surgery Combined with Empathic Nursing on Perioperative Complication Prevention and Postoperative Recovery of Gynecological Malignant Tumor Patients" was retracted in 2023. Reasons: signs of a paper mill; suspected computer-generated content; unreliable results or conclusions; concerns about the data.

## 2. Materials and Methods

### 2.1. General Data

A total of 180 patients with gynecological malignant tumor treated by surgery in our hospital from September 2018 to October 2021 were selected and randomly divided into three groups: group A, group B, and group C by random number table method, with 60 patients in each group. In group A, the age was 34-69 years old, with an average of 59.22 ± 5.86 years old. Types of diseases are as follows: 24 cases of cervical cancer, 11 cases of ovarian cancer, 14 cases of endometrial cancer, and 11 cases of fallopian tube cancer. Marital status is as follows: 55 cases of married and 5 cases of widowed or divorced. Education is as follows: 21 cases of junior college or above, 24 cases of senior high school or technical secondary school, and 15 cases of junior high school or below. In group B, the age was 33-71 years old, with an average of 58.77 ± 6.74 years old. Types of diseases are as follows: 23 cases of cervical cancer, 12 cases of ovarian cancer, 13 cases of endometrial cancer, and 12 cases of fallopian tube cancer. Marital status is as follows: 56 cases of married and 4 cases of widowed or divorced. Education is as follows: 19 cases of junior college or above, 27 cases of senior high school or technical secondary school, and 14 cases of junior high school or below. In Group C, the age was 36-70 years old, with an average of 58.25 ± 6.67 years old. Types of diseases are as follows: 25 cases of cervical cancer, 12 cases of ovarian cancer, 13 cases of endometrial cancer, and 10 cases of fallopian tube cancer. Marital status is as follows 53 cases of married and 7 cases of widowed or divorced. Education is as follows: 22 cases of junior college or above, 23 cases of senior high school or technical secondary school, and 15 cases of junior high school or below. The general data of the three groups were comparable (*P* > 0.05).

### 2.2. Inclusion and Exclusion Criteria

Inclusion criteria are as follows: (1) those who were diagnosed as gynecological malignant tumor by pathology and received surgical treatment in our hospital, (2) age ≥ 18, (3) the patient's vital signs are stable, (4) approved by the Ethics Committee of the hospital, and (5) informed consent of patients and their families. Exclusion criteria are as follows: (1) patients who were unaware of their cancer; (2) patients with previous mental illness, substance dependence, or consciousness disorder; (3) patients combined with visual disorders, aphasia, attention disorders, and communication disorders; (4) patients with defects in understanding and expression; (5) patients who were undergoing any form of psychological treatment; and (6) patients with central nervous disorder caused by trauma.

The article "Effects of the Concept of Fast-Track Surgery Combined with Empathic Nursing on Perioperative Complication Prevention and Postoperative Recovery of Gynecological Malignant Tumor Patients" was retracted in 2023. Reasons: signs of a paper mill; suspected computer-generated content; unreliable results or conclusions; concerns about the data.

### 2.3. Methods Group

A was given FTS concept combined with empathic nursing intervention, group B was given FTS concept intervention, and group C was given routine nursing intervention.

#### 2.3.1. Group C

Group C was given routine nursing intervention. (1) Preoperative: the individual situation of patients was assessed after enrollment, and the risks and knowledge associated with surgery were informed before the surgery. Solid and liquid foods were forbidden 8-12 h before surgery. Mechanical bowel preparation was routinely given before surgery. Skin preparation was performed at the operative site 1 d before surgery. Oral intestinal antibiotics were not given, and antithrombotic and analgesic sedation were not prophylactically given. (2) Intraoperative: no heat preservation measures were taken during the operation. Intravenous infusion liquid and rinse liquid at room temperature were used. (3) Postoperative: foods and water were routinely forbidden. After the recovery of anal exhaust and intestinal function, the food was transitioned from a small amount of fluid and half fluid to full fluid, half fluid, and soft food gradually according to the doctor's advice. Catheter drainage tube was indwelled and removed according to the condition. Analgesics were given as needed after operation (analgesic therapy was given when pain occurred). Patients and their families were encouraged and guided to do passive and active activities in bed, which is not mandatory.

#### 2.3.2. Group B

TFS concept intervention was given in group B. (1) Preoperative: disease counseling, education, and preoperative psychological counseling were given. After enrollment, the individual situation of the patients was evaluated, and the patients, their families, and caregivers were informed of the possible situation and corresponding coping methods in each stage of rapid recovery, and health education was given according to the individual situation of the patients. Oral solid diet was forbidden 6 h before anesthesia, and fluid diet was forbidden 2 h before anesthesia. Mechanical bowel preparation is not recommended before surgery, and short-range bowel preparation can be given when necessary. Oral intestinal antibiotics and antithrombotic drugs were prophylactically administered 1 to 3 days before surgery. (2) Intraoperative: the patient's intravenous infusion and rinse solution were warmed (the body temperature was maintained at 37 ± 0.3°C), and thermal insulation measures were continued after the operation to ensure that the patient's body temperature was above 36°C when leaving the operating room.(3) Postoperative: it is recommended that patients receive early enteral nutrition after surgery, with fluid intake on the day after surgery and normal oral intake on the first day after surgery. After anesthesia recovery, oral wetting, chewing gum, and “false feeding” therapy was adopted to promote gastrointestinal function recovery. Patients with stable vital signs could drink water immediately after awakening from anesthesia and start the dietary transition within 24 h after surgery. If the patient can meet the needs of oral nutrition, intravenous replenishment of fluid nutrition was stopped within 24 h after surgery. The patient was required to turn over and move his limbs on the first day after surgery, and the patient was encouraged to get out of bed 24 h after surgery, with the amount of activity gradually increasing. Patients and their family members were informed to reduce the times of manually pressing the analgesic pump as much as possible, and the analgesic pump using was stopped within 48 h after operation.  Table 1.

The article "Effects of the Concept of Fast-Track Surgery Combined with Empathic Nursing on Perioperative Complication Prevention and Postoperative Recovery of Gynecological Malignant Tumor Patients" was retracted in 2023. Reasons: signs of a paper mill; suspected computer-generated content; unreliable results or conclusions; concerns about the data.

#### 2.3.3. Group A

The concept of FTS concept intervention combined with empathic nursing was given in group A. The FTS concept intervention was the same as group B, and empathic nursing intervention was added on the basis of group B. The specific intervention measures were as follows: (1) admission stage: patients were often admitted with a strong sense of fear and physical and mental difficulties. We should try our best to help patients to stabilize their emotions and support them according to their personal characteristics, with explanation and comfort as priority. Through communication with patients and their families, we knew their work and life status, actively listened to patients' ideas, and patiently understood patients' psychological demands. According to their language and body movements, we analyzed their different psychology, gave psychological and physiological help, and shorten the distance between nurses and patients. We helped them adapt to the hospitalization environment and made them actively cooperate with treatment and nursing work and establish a positive and correct concept. (2) Preoperative stage: patients were inspired to remove psychological obstacles and enhance the courage to fight diseases. While explaining the treatment methods, successful cases were listed to enhance patients' confidence, provide them with a comfortable environment, reduce external adverse stimulation, avoid emotional excitement, and convey the empathy of nursing staff to patients. Patients were guided to produce correct emotional cognition and realize the sincere attitude of nursing staff, and the emotional needs of patients were deeply understood. (3) Postoperative stage: medical staff supported and comforted patients with professional knowledge, helped patients get rid of concerns, and understood patients' bad psychological emotions. The staff should patiently explain the confusion of patients, guide them to face the bad psychology with a series of methods including meditation and relaxation, listen to patients, provide them with opportunities to vent their psychological pressure, and guide them to establish a positive attitude towards life.(4) Family participation and social support: cooperation from spouse or other family members should be sought, a good job in psychological counseling of relatives should be done, so that they can fully understand patients, and give them meticulous care and full sense of security in life, playing a strong role in family support. Spouse of the patient was guided to comfort the patient through a series of ways such as encouragement, listening, persuasion, and touch based on the actual situation, spend time to accompany the patient more, and emphasize the important family status of the patient, so as to improve the patient's sense of presence and resolve bad emotions. In addition to playing a supportive role of family members, medical staff organized patient communication meetings, invited patients with similar symptoms to participate, and arranged patients with better treatment effect to introduce personal experience and popularize experience. Patients encouraged each other and gave play to the peer effect, creating a better social support atmosphere.

The article "Effects of the Concept of Fast-Track Surgery Combined with Empathic Nursing on Perioperative Complication Prevention and Postoperative Recovery of Gynecological Malignant Tumor Patients" was retracted in 2023. Reasons: signs of a paper mill; suspected computer-generated content; unreliable results or conclusions; concerns about the data.

### 2.4. Observation Indicators

(1) Preoperative blood pressure and heart rate and postoperative recovery indicator levels: blood pressure and heart rate levels at admission and 30 min before surgery were compared between the two groups. The time of first anal exhaust, time of first defecation, time of getting out of bed, and length of postoperative hospital stay were compared between the two groups. (2) Postoperative complications: the incidence of postoperative abdominal distension, poor incision healing, lymphatic cyst, urinary retention, lower limb venous thrombosis, and other complications were compared between the two groups. (3) Negative emotions: Self-rating Anxiety Scale/Self-rating Depression Scale (SAS/SDS) [12, 13] was used to evaluate patients' negative emotions before and after intervention. There were 20 items in the scale, and the score of each item was 1-4 points, including 9 positive items and 11 negative items. The total score = scale score × 1.25.SAS ≥ 50 and SDS ≥ 53, respectively, indicated the existence of anxiety or depression, and the higher the score, the more serious the negative emotion. Pain score was evaluated by pain intensity scale, 0: no pain; 1~3 points: indicates mild pain, but does not affect sleep state; 4-6 points: patients have moderate pain, and sleep status is affected; 7~10 points: the patient has severe pain, which has a serious impact on sleep.

The article "Effects of the Concept of Fast-Track Surgery Combined with Empathic Nursing on Perioperative Complication Prevention and Postoperative Recovery of Gynecological Malignant Tumor Patients" was retracted in 2023. Reasons: signs of a paper mill; suspected computer-generated content; unreliable results or conclusions; concerns about the data.

### 2.5. Statistical Method

SPSS21.0 was used to analyze the data. Measurement data were expressed by $\bar{X}\pm S$. The measurement data followed normal distribution and met homogeneity of variance. Independent sample *T* test was used for intergroup comparison, and one-way ANOVA was used for intergroup comparison. Enumeration data were expressed by number of cases or percentage, and chi-square test was used for comparison between groups. *P* < 0.05 indicated statistically significant difference.

## 3. Results

### 3.1. Comparison of Preoperative Blood Pressure and Heart Rate among the Three Groups

There were no significant differences in blood pressure and heart rate among the three groups before admission (*P* > 0.05). Systolic blood pressure, diastolic blood pressure, and heart rate of the three groups increased 30 min before operation compared with that of the admission, and the blood pressure and heart rate of group C were higher than those of groups A and B, and the blood pressure and heart rate of group A were the lowest (*P* < 0.05) Table 2.

### 3.2. Comparison of Postoperative Recovery Indicators among Three Groups

The time of first anal exhaust, time of first defecation, time of getting out of bed, and postoperative hospital stay in groups A and B were shorter than those in group C (all *P* < 0.05, Table 3).

### 3.3. Comparison of Postoperative Complications among the Three Groups

The incidence of postoperative complications in groups A and B was 8.33% and 8.33%, respectively, lower than 23.33% in group C (both *P* < 0.05, Table 4).

### 3.4. Comparison of Pain Scores among the Three Groups

There was no significant difference in preoperative pain scores among the three groups (*P* > 0.05). There was no statistical significance in the pain scores of the three groups after operation (*P* > 0.05). There was no significant difference in pain scores before and after surgery among the three groups (Table 5, *P* > 0.05).

### 3.5. Comparison of Psychological States among the Three Groups

The negative emotions of the three groups before intervention were comparable (*P* > 0.05). After intervention, psychological distress, SAS, and SDS scores of the three groups were lower than those before intervention, and group A was lower than group B and group C (all *P* < 0.05, Table 6).

The article "Effects of the Concept of Fast-Track Surgery Combined with Empathic Nursing on Perioperative Complication Prevention and Postoperative Recovery of Gynecological Malignant Tumor Patients" was retracted in 2023. Reasons: signs of a paper mill; suspected computer-generated content; unreliable results or conclusions; concerns about the data.

## 4. Discussion

According to the data of China's national tumor registry released in 2016, cervical cancer, endometrial cancer, and ovarian cancer all rank among the top 10 female malignant tumors [14, 15]. Clinically, middle-aged and elderly women are the group with high incidence of gynecological malignant tumors. Relatively speaking, middle-aged and elderly women have weaker constitution and slower postoperative recovery [16].

In recent years, the nursing mode in China has gradually changed from “disease-centered” to “patient-centered” [17]. Based on gynecological malignant tumor surgery and psychological characteristics of patients, targeted nursing intervention is of great significance to postoperative rehabilitation of patients [18]. The FTS concept is based on the principle of body stress, and its basic principle is reducing body stress and surgical complications. Based on evidence-based medical evidence, a series of perioperative management measures are optimized and integrated to accelerate the recovery process of patients [19, 20]. Traditional nursing intervention is often the experience intervention of medical staff. Patients with low service satisfaction are more likely to have physical symptoms aggravated by their own emotional experience and poor mood. Empathy is a platform for communication between nurses and patients, as well as a starting point for establishing a good nurse-patient relationship [21]. Compared with conventional nursing forms, empathic nursing enables nursing staff to fully understand the basic needs of patients in the way of perspective-taking, improve nursing measures according to the needs of patients, and carry out comprehensive nursing intervention from the aspects of patients, wards, treatment, and nursing [22].

The operation itself is a serious psychological and physiological stress, coupled with the lack of knowledge of surgery and anesthesia, and preoperative adverse psychological is common in patients. Chang et al. [23] showed that psychological stress will directly affect the physiological activities of patients, mainly manifested by sympathetic nerve-adrenal medulla excitation and hypothalamus-pituitary-adrenal cortex secretion (increased blood pressure, accelerated heart rate, etc.). As a result, anxiety hypertension and abnormal heart rate and behavior (irritability, poor cooperation with medical staff, etc.) occurred before surgery, which seriously affected perioperative preparation, treatment, and postoperative rehabilitation. In the present study, blood pressure and heart rate levels 30 min before surgery in the three groups were compared, and the results showed that the blood pressure and heart rate levels of group A were lower than those of group B, and that of group B was lower than that of group C. This indicated that the concept of FTS combined with empathic nursing was conducive to improving the preoperative stress response of patients, enabling them to receive surgery in a better state with relatively stable vital signs. For one thing, the FTS concept emphasizes the preoperative disease education for patients, so that they have a clear understanding of the treatment and nursing content. Patients can actively participate in the self-care and to a certain extent and alleviate the anxiety of patients. For another thing, empathic nursing carries out targeted psychological intervention according to the different psychology of patients in different stages. Medical staff patiently listen to patients' needs, communicate with patients, give patients comfort, encouragement, and support, dredge bad mood, meet their psychological needs, and improve preoperative stress. The postoperative recovery of the two groups was further compared. In this study, the first postoperative anal exhaust time and first defecation time of patients in group A and group B were shorter than those in group C. Exhaust and defecation time is an objective indicator of postoperative gastrointestinal function recovery. In this study, the key reason for the shortening of postoperative exhaust and defecation time of patients in group A and group B lies in the good preparation of gastrointestinal tract based on TFS concept during perioperative period. Before operation, mechanical enema was avoided to prevent intestinal flora imbalance, dehydration, and electrolyte balance disorder. After operation, early oral diet promoted the recovery of postoperative intestinal function under the regulation of gastrointestinal neuroendocrine. In addition, in this study, the ambulation time and postoperative hospitalization time of groups A and B were shorter than those of group B. Based on the actual situation of patients, TFS concept actively carries out a number of preoperative, intraoperative, and postoperative measures to reduce patients' discomfort, strengthen postoperative rehabilitation, carry out early ambulation, strengthen postoperative enteral nutrition, and promote perioperative recovery of patients. Liu [24] showed that TFS concept can significantly reduce pain and the risk of complications in patients with cervical cancer. The current study compared the incidence of perioperative complications among the three groups, and the results showed that the incidence of postoperative complications in group A and group B was lower than that in group C. This indicated that the implementation of TFS concept was beneficial to reduce the risk of postoperative complications of gynecological malignant tumors, which is consistent with the above results. Routine perioperative intervention of mechanical intestinal preparation increases the risk of postoperative peritoneal infection and anastomotic fistula. TFS concept advocates that patient get out of bed early to reduce the risk of pulmonary complications, and patients' muscle strength and tissue oxygen supply are strengthened. Early enteral nutrition also accelerates the recovery of gastrointestinal function and reduces the risk of intestinal obstruction. At the same time, TFS concept also reduces the incidence of urinary infection and urinary retention to a certain extent and prevents the formation of deep venous thrombosis in lower limbs.

The article "Effects of the Concept of Fast-Track Surgery Combined with Empathic Nursing on Perioperative Complication Prevention and Postoperative Recovery of Gynecological Malignant Tumor Patients" was retracted in 2023. Reasons: signs of a paper mill; suspected computer-generated content; unreliable results or conclusions; concerns about the data.

Perez-Fuentes et al. [25] applied empathy in nursing work, and patients' physical anxiety and depression were significantly improved after intervention. The results of the present study showed that the anxiety and depression mood score of group A was lower than that of group B and group C after intervention, which was consistent with the above research results. The implementation of empathic nursing intervention in group A treated patients' bad psychological emotions with professional skills and services and showed full understanding and respect to patients. In addition to taking into account the physical factors of the patient, we also pay attention to the mental aspects of the patient. We encouraged patients to look at problems with a positive perspective, change their psychological state, emphasize the joint support and intervention of their spouses and other family members, and provide corresponding dietary care, emotional comfort, physical touch, and rehabilitation care. This enabled patients to fully feel the existence of their families and get enough psychological support, which improved their anxiety, depression, and other emotions and relieved adverse psychological problems. At the same time, while helping patients correctly understand the disease, empathic nursing provided corresponding social support to patients, set up communication meetings, encouraged patients to comfort and help each other, and improved patients' confidence. The combined concept of empathy can further improve the effect of negative emotion. The reason may be that the concept of empathy thinks from the perspective of the patient and correctly understands the feedback of the patient by feeling the psychological and emotional changes of the patient. The deficiency of this study is that there were significant differences in surgical methods and perioperative reactions among patients with different tumor types and stages. This study did not discuss the application value of FTS concept combined with empathic nursing. In the follow-up study, the sample size will be further expanded and classified discussion and analysis will be carried out.

The article "Effects of the Concept of Fast-Track Surgery Combined with Empathic Nursing on Perioperative Complication Prevention and Postoperative Recovery of Gynecological Malignant Tumor Patients" was retracted in 2023. Reasons: signs of a paper mill; suspected computer-generated content; unreliable results or conclusions; concerns about the data.

In conclusion, FTS concept combined with empathic nursing was beneficial to reduce the stress response of patients with gynecological malignant tumor before surgery, reduce the risk of postoperative complications, improve patients' negative emotions, strengthen the psychological response to the disease, and speed up the recovery process of patients.

## Figures and Tables

**Table 1:** Comparison of items between routine intervention and FTS concept intervention.

Item	Routine intervention	FTS concept intervention
Preoperative	(1) Routine preoperative education (2) Abstain from water for 8-12 h before surgery (3) Mechanical bowel preparation	(1) Preoperative education and health education for specific diseases (2) Abstain from solid food for 6 h before surgery, liquid diets for 2 h (3) Canceling mechanical bowel preparation (4) Preoperative prophylactic administration of antibiotics and antithrombotic drugs
Intraoperative	(1) No insulation	(1) Prevention of hypothermia, heat preservation measures
Postoperative	(1) Diet after anal exhaust (2) Encouraging and guiding patients and their families to do passive and active activities in bed, not mandatory (3) Analgesic pump installing, which was stopped within 48 h after operation	(1) Receiving early enteral nutrition (2) Encouraging and urging patients to get out of bed 24 h after the operation (3) Analgesic pump installing, informing patients and their families to reduce the manual pressing times of the analgesic pump as much as possible, and stopping using it within 48 h after operation

**Table 2:** Comparison of preoperative blood pressure and heart rate among the three groups ($\bar{X}\pm S$).

Group	Time	Systolic blood pressure (Hg)	Diastolic blood pressure (mmHg)	Heart rate (times/min)
Group A (*n* = 60)	At admission	112.47 ± 4.32	74.12 ± 3.64	75.42 ± 7.88
	30 min before surgery	117.47 ± 3.49^①②③^	76.97 ± 3.20^①②③^	82.03 ± 5.97^①②③^
Group B (*n* = 60)	At admission	112.32 ± 5.48	74.27 ± 3.31	75.85 ± 6.84
	30 min before surgery	120.67 ± 4.13^①②^	78.98 ± 2.70^①②^	85.85 ± 5.22^①②^
Group C (*n* = 60)	At admission	112.82 ± 5.28	74.28 ± 2.98	76.52 ± 5.83
	30 min before surgery	122.87 ± 4.44^①^	82.77 ± 2.08^①^	89.03 ± 4.66^①^

Note: Compared with before intervention, ^①^*P* < 0.05; compared with group C, ^②^*P* < 0.05; compared with group B, ^③^*P* < 0.05.

The article "Effects of the Concept of Fast-Track Surgery Combined with Empathic Nursing on Perioperative Complication Prevention and Postoperative Recovery of Gynecological Malignant Tumor Patients" was retracted in 2023. Reasons: signs of a paper mill; suspected computer-generated content; unreliable results or conclusions; concerns about the data.

**Table 3:** Comparison of postoperative recovery indicators among three groups.

Group	Time of first anal exhaust (h)	Time of first defecation (h)	Out of bed time (h)	Postoperative hospital stay (d)
Group A (*n* = 60)	23.13 ± 2.43^①^	42.32 ± 6.25^①^	20.00 ± 4.59^①^	7.62 ± 0.97^①^
Group B (*n* = 60)	23.17 ± 2.94^①^	42.58 ± 6.03^①^	21.65 ± 4.55^①^	7.95 ± 1.24^①^
Group C (*n* = 60)	31.55 ± 4.72	56.12 ± 6.18	50.17 ± 5.65	10.38 ± 1.34

Note: Compared with group C, ^①^*P* < 0.05.

**Table 4:** Comparison of postoperative complications among the three groups.

Group	Infection	Poor incision healing	Lymphocyst	Urinary retention	Thrombus of lower extremity veins	Overall incidence n (%)
Group A (*n* = 60)	1	2	2	0	0	5 (8.33)^①^
Group B (*n* = 60)	3	1	1	0	0	5 (8.33)^①^
Group C (*n* = 60)	3	3	4	3	1	(23.33)

Note: Compared with group C, ^①^*P* < 0.05.

**Table 5:** Comparison of pain scores among the three groups.

Group	Time	Pain score
Group A (*n* = 60)	Before intervention	4.10 ± 1.03
	After intervention	3.88 ± 0.94
Group B (*n* = 60)	Before intervention	4.93 ± 0.43
	After intervention	4.17 ± 0.51
Group C (*n* = 60)	Before intervention	4.28 ± 1.03
	After intervention	4.05 ± 0.65

Note: Compared with before intervention, ^①^*P* < 0.05; compared with group C, ^②^*P* < 0.05; compared with group B, ^③^*P* < 0.05.

**Table 6:** Comparison of psychological states between the three groups ($\bar{X}\pm S$, point).

Group	Time	SAS 25-100	SDS
Group A (*n* = 60)	Before intervention	48.57 ± 4.83	47.80 ± 3.48
	After intervention	38.28 ± 3.94^①②③^	35.30 ± 4.03^①②③^
Group B (*n* = 60)	Before intervention	47.93 ± 5.43	47.32 ± 4.80
	After intervention	42.17 ± 5.51^①②^	40.00 ± 5.24^①②^
Group C (*n* = 60)	Before intervention	48.28 ± 5.03	48.18 ± 5.10
	After intervention	43.05 ± 4.65^①^	40.52 ± 5.28^①^

Note: Compared with before intervention, ^①^*P* < 0.05; compared with group C, ^②^*P* < 0.05; compared with group B, ^③^*P* < 0.05.

## Data Availability

The labeled dataset used to support the findings of this study are available from the corresponding author upon request.
